# Multifactor Logistic Analysis to Explore the Risk Factors of Safety Risks in the Transport of Critically Ill Patients with ICU and the Improvement of Nursing Strategies

This article has been retracted.

**DOI:** 10.1155/2022/3330667

**Published:** 2022-05-14

**Authors:** Zhenyu Zhang, Hui Qu, Wei Gong

**Affiliations:** ^1^Department of Intensive Care Unit (Eastern), Yantai Yuhuangding Hospital, Yantai 264000, Shandong Province, China; ^2^Department of Intensive Care Unit (Western), Yantai Yuhuangding Hospital, Yantai 264000, Shandong Province, China; ^3^Department of Cardiac Intensive Care Unit, Yantai Yuhuangding Hospital, Yantai 264000, Shandong Province, China

## Abstract

**Objective:**

Multivariate logistic analysis was employed to explore the risk factors of safety risks in the transport of critically ill patients with ICU and the improvement of nursing strategies.

**Methods:**

Two hundred critical transport patients with ICU treated in our hospital from January 2019 to April 2021 were enrolled. According to the occurrence of unsafe events in transit, the patients were assigned to the control group (165 cases without unsafe events, *n* = 165) and the study group (35 cases with safety incidents, *n* = 35). Multivariate logistic analysis was employed to explore the risk factors of safety risks in the transport of critically ill patients with ICU and to enhance nursing strategies.

**Results:**

(1) General data of the subjects: among the 200 critically ill patients with ICU who needed in-hospital transport, the age ranged from 18 to 85 years with an average age of 52.48 ± 3.31, including 89 males and 111 females. There were 35 cases of gastrointestinal bleeding, 16 cases of respiratory failure, 23 cases of heart failure, 43 cases of myocardial infarction, 26 cases of cerebrovascular accident, 14 cases of ectopic pregnancy, 25 cases of severe injury, and 18 cases of mechanical ventilation. There were 35 cases in the study group with accidents and 45 cases in group B without accidents. (2) Among the 200 patients, 35 patients had complications during the transit process in the intermediate people's court, with an incidence rate of 17.5%. It included blood pressure fluctuation (*n* = 6), artificial airway obstruction (*n* = 6), decrease in blood oxygen saturation (*n* = 10), dyspnea (*n* = 5), fall pain (*n* = 3), elevated intracranial pressure (*n* = 2), and other factors (*n* = 3). There exhibited no significant difference in blood oxygen saturation at each time point during transport (*P* > 0.05). There exhibited no significant difference in SpO_2_ before transport. The comparison of 5 min and 10 min blood oxygen saturation during transit in the study group was lower compared to the control group (*P* < 0.05). (3) In a univariate analysis of safety risks for critically ill ICU patients, home escorts did not show significant differences in hospital transport for critically ill ICU patients (*P* > 0.05). There were significant differences in terms of age, patient's condition, transport escort, auxiliary ventilation, means of transport, uncarried drugs and goods, and carrying pipeline (*P* < 0.05). The results of multivariate logistic regression analysis indicated that age, patient's condition, transport escort, auxiliary ventilation, means of transport, uncarried drugs and goods, and carrying pipeline were the risk factors affecting the safe transport of critically ill patients (*P* < 0.05).

**Conclusion:**

Age, patient's condition, transport escort, auxiliary ventilation, means of transport, uncarried drugs and goods, and carrying pipeline are the independent risk factors that affect the safe transport of emergency or ICU critically ill patients. Therefore, in order to reduce the risk of transshipment, we must enhance the safety awareness of escorts, strengthen the management and training of escorts, promote rules and regulations, and formulate dangerous plans, so as to eliminate the occurrence of unsafe factors.

## 1. Introduction

In-hospital transport refers to the transfer of patients between different departments of the same medical unit, and its main task is to carry out related examination and treatment, as well as the transfer of patients when they are admitted to other departments of the same hospital [1]. In order to make patients get more comprehensive diagnosis and treatment and restore their health as soon as possible, the necessary transport is indispensable in the clinical diagnosis and treatment of patients. Emergency ICU patients' condition changes rapidly, so it is difficult to transport and the risk of transport is high [2]. The transportation safety of critically ill patients has always been a hot topic recently. In 2015, American medical institutions listed “patient transport” as one of the top 10 patient safety issues to be concerned about [3]. Although the transit time ranges from a few minutes to several hours, it may bring about all kinds of side effects due to the limitations of medical conditions, alterations in the environment, uneven transport and escort personnel, different conditions, and poor stability [4]. The study reported that the incidence of adverse events in transit was 31.3%, even as high as 70% [5]. Critical patients in hospital transport are prone to adverse reactions such as change in blood pressure, decrease of SpO_2_, arrhythmia, and change of consciousness, among which the decrease of SpO_2_ is the most common [6]. Hypoxia is bound to affect the metabolism of patients and delay recovery of patients; the decrease of SpO_2_ can aggravate the oxidative damage of red blood cells, resulting in a vicious circle of hypoxia, thus affecting the recovery of patients [7].

The side effects of the patients during the transfer may be related to the patient's condition, the excellent transfer equipment, the ability of the transfer personnel or the communication between the teams, the preparation before the transfer, and the monitoring during the transfer [8]. According to reports of adverse events during in-hospital transport, patients had different types of complications during in-hospital transport, of which 42.4% of the complications were related to hypoxia [9]. Some scholars reported that during the transfer of surgical patients to the ward, about 30% to 50% of patients developed hypoxemia after operation. About 87% of transport patients need different levels of oxygen supply during the transport, and 38% of patients have changes in SpO_2_ during the transport. Due to the degenerative diseases of the respiratory system and the decline of respiratory function in elderly patients, it is easy to cause potential physiological hypoxemia, that is, senile hypoxemia [10]. Respiratory disorders caused by bronchial and pulmonary lesions in patients with respiratory diseases may lead to hypoxia during transport, resulting in the decrease of SpO_2_ in patients. In addition, some patients can maintain their normal blood oxygen saturation during rest, but hypoxemia often occurs during walking, sleeping, or exercise [11]. Changes in position during transfer and movement may lead to changes in breathing patterns and psychological changes, resulting in dizziness, palpitations, shortness of breath, and other symptoms [12]. In order to ensure that oxygen therapy patients absorb oxygen effectively during transport, an oxygen bag is the most commonly employed clinical oxygen supply device, which is the most widely employed. Some scholars have indicated that transshipment personnel are one of the risk factors of unsafe transshipment during in-hospital transshipment. The lack of communication among team members makes the work inefficient, and the transfer time is prolonged, which may lead to adverse events [13]. The adverse events during transport mainly included hypoxemia, airway obstruction, displacement or prolapse of endotracheal catheter, shedding of arteriovenous lines, severe fluctuation of hemodynamics, increased intracranial pressure, hemorrhage, and even cardiorespiratory arrest, sudden death, and other serious adverse consequences [14]. Therefore, it is of great significance to screen the risk factors of safe transport between hospitals and take effective preventive measures to avoid the occurrence of the accidents, reduce the mortality during transport, improve the prognosis of patients, and reduce medical accidents. At present, the studies on the transport of critically ill patients are mostly focused on the complications that may occur during the transport of critically ill patients, but there is no further analysis and research on the risk factors of transport safety of critically ill patients in ICU. In this regard, the purpose of this study is to explore the risk factors of safety risks in the transport of critically ill patients with ICU and put forward targeted intervention countermeasures, so as to reduce the incidence of safety risks in the transport of critically ill patients.

## 2. Patients and Methods

### 2.1. General Information

Two hundred critical transport patients with ICU in our hospital from January 2019 to April 2021 were enrolled. According to the occurrence of unsafe events in transit, the patients were assigned to the control group (165 cases without unsafe events, *n* = 165) and the study group (35 cases with safety incidents, *n* = 35). This study was permitted by the Medical Ethics Association of our hospital, and all patients signed informed consent.

*Selection criteria*: (1) patient's age ≥ 18 years; (2) patients' vital signs are relatively stable under the condition of oxygen supply in emergency ICU center and SpO_2_ ≥ 94%; and (3) patients who continue oxygen therapy according to doctor's advice during transport.

*Exclusion criteria*: (1) restless patients; (2) patients who died during transit.

### 2.2. Treatment Methods

The following data were collected by consulting the evaluation form of in-hospital transfer in the department: (1) including general data: sex, body weight, age, time of seeing a doctor, preliminary diagnosis, and whether the family members were accompanied or not and (2) pretransport assessment: vital signs: body temperature, pulse, respiratory rate, blood pressure, consciousness, and blood oxygen saturation; patient's condition: type I, class II, class III, class IV, and class V. According to the Canadian preexamination triage (CTAS) standard, the patients are assigned to five categories according to the severity of the disease; artificial airway: whether mechanical ventilation is needed; deep vein catheterization: yes or no; establishment of vein: yes or no; posture: comfortable and passive; (3) preparation before transport: auxiliary nurses, first-class nurses, second-class nurses, and doctors; patients carrying drugs and goods; carrying pipelines; and purpose of transport; transport tools: flat car, wheelchair; (4) destination assessment: vital sign monitoring indicators: body temperature, pulse, respiratory rate, blood pressure, consciousness, and blood oxygen saturation; (5) recording of accidents during transport: bed rest, interruption of oxygen supply, blockage or detachment of infusion tube and various drains, sudden drop in blood pressure, decrease in blood oxygen saturation, asphyxia, cardiac arrest, and changed consciousness; (6) time to start transfer; and (7) time to arrive at the department.

The criteria for judging accidents are as follows:

*Sudden drop in blood pressure*: (1) systolic blood pressure < 80 mmHg (1 mmHg = 0.133 kPa), (2) pulse pressure difference < 20 mmHg, and (3) systolic blood pressure in patients with original hypertension decreased by more than 30% compared with the original level. One of the blood pressures in emergency adult patients during hospital transport was recorded as a sudden drop in blood pressure.

*Asphyxia [* 15 *]*: (1) restlessness and nasal incitement, (2) blue lips and cyanosis, and (3) weak and fast pulse, decreased blood pressure, and dilated pupils. The simultaneous occurrence of the three was judged as asphyxia.

*Cardiac arrest*: diagnostic criteria include (1) loss of consciousness, (2) pulsation of carotid artery and femoral artery disappearance and heart sound disappearance, (3) sigh-like breathing which can urgently restore blood circulation and stop breathing, and (4) the light reflex of dilated pupil weakening to disappearance; meanwhile, the electrocardiogram demonstrates the following: (1) ventricular fibrillation or flutter accounts for about 91%, (2) electro-cardio-mechanical separation has wide and deformed, low-amplitude QRS frequency 20 to 30 beats per minute to produce myocardial mechanical contraction, and (3) ventricular rest is a straight line of nonelectric waves.

*Decrease of blood oxygen saturation [* 16 *]*: (1) partial pressure of arterial oxygen is less than 60 mmHg and (2) blood oxygen saturation decreases by more than 5% during transport. One of them is the decrease in blood oxygen saturation.

### 2.3. Statistical Analysis

Epidata3.0 software is adopted for double-blind data input, and the SPSS 17.0 statistical software package is employed for analysis. The measurement data of normal distribution are expressed by the mean standard deviation $\bar{x}\pm s$, the group *t*-test was adopted for the comparison of measurement data, and the chi-squared test was employed for the comparison of counting data. The above influencing factors were compared, and the risk factors with statistically significant differences were analyzed by multifactor logistic regression analysis to screen out the risk factors affecting hospital safe transport in critically ill patients with ICU. *P* < 0.05 indicates statistically significant.

## 3. Results

### 3.1. General Data of the Object of Study

First of all, we analyzed the general data of the patients. Among the 200 critically ill patients with ICU who needed hospital transfer, the age ranged from 18 to 85 years old with an average age 52.48 ± 3.31, including 89 males and 111 females. There were 35 cases of gastrointestinal bleeding, 16 cases of respiratory failure, 23 cases of heart failure, 43 cases of myocardial infarction, 26 cases of cerebrovascular accident, 14 cases of ectopic pregnancy, 25 cases of severe injury, and 18 cases of mechanical ventilation. There were 35 cases in the study group with accidents and 45 cases in group B without accidents. All the data results are indicated in Figure 1.

### 3.2. Occurrence of Complications during Transport

Secondly, we analyzed the occurrence of complications in the process of transport. Among the 200 patients, 35 patients had complications in the process of transport in the intermediate people's court, with an incidence of 17.5%. It included blood pressure fluctuation in 6 cases, artificial airway obstruction in 6 cases, decrease of blood oxygen saturation in 10 cases, dyspnea in 5 cases, fall injury in 3 cases, elevated intracranial pressure in 2 cases, and other factors in 3 cases. The specific occurrence of complications is indicated in Figure 2.

### 3.3. Blood Oxygen Saturation at Different Time Points during Transport

Thirdly, we compared the blood oxygen saturation of the patients at each time point during transport. There exhibited no significant difference in SpO_2_ before transport (*P* > 0.05). The comparison of 5 min and 10 min and blood oxygen saturation during transit in the study group was lower compared to the control group (*P* < 0.05). All the data results are indicated in Table 1.

### 3.4. Single Factor Analysis of Safety Risks in Critically Ill Patients with ICU during Transport

Then, we conducted a univariate analysis of the safety risks in critically ill patients with ICU. The results indicated that there exhibited no significant difference in family escort in the hospital transport of critically ill patients with ICU (*P* > 0.05). There were significant differences in terms of age, patient's condition, transport escort, auxiliary ventilation, means of transport, uncarried drugs and goods, and carrying pipeline in critically ill patients with ICU (*P* < 0.05). The specific results are indicated in Table 2.

### 3.5. Results of Multivariate Logistic Regression Analysis

Finally, we carried out multifactor logistic regression analysis on the factors affecting the in-hospital safe transport of critically ill patients with ICU. The factors affecting the in-hospital safe transport of critically ill patients with ICU were compared. The detailed values of each factor are indicated in Table 3, and the multifactor logistic regression analysis is carried out. The results indicated that age, patient's condition, transport escort, auxiliary ventilation, means of transport, uncarried drugs and goods, and carrying pipeline were the risk factors affecting the safe transport of critically ill patients with ICU in hospital. The analysis results are indicated in Table 4. The difference of data was statistically significant (*P* < 0.05).

## 4. Discussion

ICU is the first choice for critically ill patients, critically ill patients need hospital transport after emergency treatment, and the purpose of transport is that patients need to be hospitalized for further treatment or related diagnostic examination [16]. Although inpatient referrals are short, the risks are present throughout the referral process [17]. The case fatality rate of critically ill patients with ICU during hospital transfer was 9.6% higher compared to usual [18]. During the hospital transfer, the accompanying personnel are uneven; the patients' conditions are different; their stability is usually poor; nurses do not receive formal first aid training, do not carry rescue drugs and articles, and lack resources; and limited monitoring equipment may lead to unsafe transfer [19]. With the sudden change of the surrounding environment, the patient's condition will change unpredictably, which poses a great threat to the patient's life [20]. The side effects during transport mainly included hypoxemia, airway obstruction, displacement or prolapse of endotracheal catheter, shedding of arteriovenous lines, severe fluctuation of hemodynamics, increased intracranial pressure, hemorrhage, and even cardiorespiratory arrest, sudden death, and other serious adverse consequences [21]. Risk factors usually include two aspects: patient factors and medical factors; the former includes patient condition factors and posture factors; the latter includes escort personnel factors, equipment and drug factors, transport tool factors, and communication and coordination factors.

During the in-hospital transfer, there can be some factors, such as unpredictable changes in illness, lack of monitoring and treatment equipment, lack or exhaustion of medical staff, and other factors, leading to malignant events during the transfer of patients in the hospital [22]. Some academics believe that pulse oximetry, blood pressure fluctuations, hypoxia, and hypotension are used as indicators to assess safe transport. The results suggest that 38.1% of patients do not comply with safe transport [23]. In the survey data of in-hospital transport of critically ill patients, it was found that the incidence of side effects related to the patient's condition was about 31%, including the circulatory system, respiratory system, digestive system, and central nervous system [24]. In other scholars' studies, respiratory and cardiac arrest may occur in patients with severe craniocerebral injury, cerebral hemorrhage, cardiac injury, pericardial tamponade, myocardial infarction, heart failure, and respiratory failure [25]. Furthermore, critically ill patients carry all kinds of pipes, such as endotracheal intubation, ventilator line, indwelling venous passage, and drainage tube [26]. Patients are irritable and unconscious, which affect the safety of hospital transportation. During the transfer period, due to the influence of various reasons, the special posture is easy to change. Special positions can lead to poor contact with instruments such as ECG monitoring, interfering with measurements, and affecting judgment of disease. It may also lead to inadequate perfusion of vital organs, especially in patients with multiple injuries, and therefore, changes in position due to exercise should be prevented. In addition, the handling process should pay more attention to the protection of patients' personal privacy and should not be carried blindly, causing psychological harm to patients. The means of transportation should be enrolled according to the specific conditions of the patients. Once improperly enrolled, not only will it easily lead to damage to the patient's neck and limbs, falling out of bed, hypoxia, shedding, or displacement of the carrying pipe but also the patient's position will easily change. As a result, the monitoring of vital signs is disturbed, which affects the accurate judgment of the patient's condition, prolongs the transfer time, and increases the risk of transport. Some scholars have also indicated that improper use of transport tools can lead to hypoxia, carrying the pipeline to fall off and shift, resulting in the occurrence of unsafe transport [27]. It is necessary to pretreat the high-risk in-hospital transshipment in advance, which is an important measure to reduce the risk level and ensure the safety of transshipment. In many nursing disputes, the vast majority of disputes do not belong to medical malpractice but do not explain clearly before transshipment, and some people do not understand and bear medical risks [28]. Therefore, after deciding on the transfer to the hospital, the doctor in charge should inform the patients and their families of the necessity and potential risks of the transfer and obtain informed consent and signature of the patients and their families.

Patient transport is an important part of medical work and the top priority of medical safety [29]. Maintaining the stability of patients' vital signs is an important prerequisite for transport safety. Proper provision of oxygen therapy can effectively ensure the stability of patients' vital signs and reduce the occurrence of clinical complications to a great extent. An excellent oxygen therapy device is an important guarantee to ensure the full absorption of oxygen by transporting patients. Clinically, there are a variety of devices used to provide oxygen therapy when transporting patients; each has its own advantages and disadvantages. This article reviews the oxygen therapy devices commonly used in clinical transport of patients. Patient transfer includes interhospital and intrahospital transfer, mainly for local hospitals due to the limitations of medical conditions, not meeting the treatment needs of special patients, and can only be transferred to higher-level hospitals for treatment [29]. In-hospital transport refers to the necessary transport process of patients between departments in the hospital, and its main task is to make a clear diagnosis and carry out relevant examinations, such as MRI, CT, X-ray examination, and surgical treatment, as well as emergency and ICU patients admitted to other departments for transport [29, 30]. In order to make patients get more comprehensive diagnosis and treatment and restore their health as soon as possible, the necessary transport is indispensable in the clinical diagnosis and treatment of patients. However, in the process of transport, due to the limitations of medical conditions and sudden changes in the environment, all kinds of medical adverse events may occur during the transfer of patients [30]. In the latest concept of patient transport, it is mentioned that the main purpose of all transport is to maintain medical continuity and prevent any adverse events that may seriously affect the prognosis of patients. Only when medical and nursing staff have the necessary skills, equipped with good transport equipment, and have a well-developed transport process can they minimize the risks of transport and ensure the safety of patient transport [31].

The improved nursing strategies are as follows: (1) pretransshipment patient assessment: critically ill patients may cause great harm to patients or even cause death due to unexpected events for different reasons in the course of transportation. Before the patient enters the emergency department for rescue, it is necessary to evaluate the patient to understand the patient's vital signs and life status. The main contents of the assessment include patients' awareness, vital signs, medication, respiratory tract conditions, and possible safety risks in the process of transport. In the process of patient assessment, it is necessary to comprehensively consider the situation of the patient and the situation of the emergency department, as well as the risks that may exist in the process of transportation; (2) pretransshipment nursing preparation: in order to ensure the safety of patients in the process of transshipment, full preparation should be made before transshipment. The main operations before the transfer of critically ill patients in the emergency department of the hospital include nurse preparation, that is, the selection of nurses who have experience and skills and who have a better understanding of the patient's illness and can face emergencies; route preparation, according to the confirmation of the department to which the patient needs to be transferred and according to the route from the emergency department to the department, it is appropriate to plan according to the route from the emergency department to the department, so as to achieve safe transfer as soon as possible. In item preparation, in the process of transshipment, nurses need to fully prepare drugs, articles, transshipment oxygen cylinders, detectors, and other instruments to ensure that the items in the transshipment process are in place. Patient preparation: for some patients in coma or extremely critical conditions, it is necessary to use a ventilator or other detectors for the patient according to the patient's vital signs, and meanwhile, in order to prevent the patient from falling from the transfer bed, it is necessary to give the patient a relatively comfortable state and fixed treatment, which should ensure not only safety but also speed and patient comfort in the process of transport. The family members of the patients are prepared to communicate with the family members of the patients in advance before the transfer, including matters needing attention, the location of the transfer, and the preparation of the transfer. (3) Nursing work during transit: pay attention to the details in the process of safe transport. If the patient is awake, he needs to communicate with the patient and ask the patient if he feels any discomfort [32]. If the patient is in a coma or unable to express, pay close attention to the patient, including posture, status, and vital signs. In the process of transport, it is necessary to keep the transfer process as smooth and fast as possible to avoid oscillation and affect patients. Keep the patient's head in front of the escort and keep the head high when going uphill. For example, in the process of transport in winter, if you need to go through the outdoor environment, you should pay attention to keep the patients warm and be exposed to the wind, so as to prevent them from getting worse or causing typhoid fever [33]. Paying attention to the details of the disease in the process of transport, nurses need to closely observe the vital signs and status of the patient, including the patient's mind, heart rate, blood pressure, blood oxygen saturation, connection between trachea and respirator, and infusion needles. If the patient also needs to pass through the tube such as oxygen infusion or infusion in the process of transport, the pipeline needs to be observed to prevent blockage and reflux. For the safety details of the inspection process when the patient needs to carry out the examination, the patient needs to be protected to prevent sudden risks. If the patient is still in a coma, the patient needs to be fixed and photographed to prevent a fall. (4) Safety nursing after transfer: after arriving at the destination, it is necessary to carefully complete the handover with the nurses in the department. The contents of handover include all kinds of related data and indicators, such as patient's consciousness, triage, pupil, vital signs, examination, infusion site, medication, pipe name, implantation depth, and oxygen flow. And the relevant nursing matters needing attention of the patients were handed over. If the patient is not accompanied by a family member, he or she also needs to help the patient hand over and place his personal belongings. After the completion of the transfer, it is necessary to count the items used in the transfer to prevent the loss of the items and affect the safe use of the transfer of other patients [34].

In summary, the age, patient's condition, transport escort, auxiliary ventilation, means of transport, uncarried drugs and articles, and carrying pipeline of ICU critically ill patients are independent risk factors that affect the safe transport of emergency patients. Therefore, in order to reduce the risk of transshipment, we must enhance the safety awareness of escorts, strengthen the management and training of escorts, promote rules and regulations, and formulate dangerous plans, so as to eliminate the occurrence of unsafe factors.

## Figures and Tables

**Figure 1:** General information of research object.

**Figure 2:** Occurrence of complications during transportation.

**Table 1:** Comparison of blood oxygen saturation between the two groups at different time points during transport $\left(\bar{x}\pm s,\%\right)$.

Group	*N*	Before transshipment	Transfer 5 min	Transfer 10 min	Reach the destination
C group	165	98.49 ± 0.31	97.39 ± 0.25	95.31 ± 1.24	93.54 ± 1.21
R group	35	98.41 ± 0.41	93.49 ± 2.45	92.59 ± 3.12	90.55 ± 3.12
*t*		1.305	20.142	8.516	9.460
*P*		>0.05	<0.01	<0.01	<0.01

**Table 2:** Single factor analysis of safety risks in critically ill patients with ICU during transport $\left(\bar{x}\pm s,n/\%\right)$.

Group	C group (*n* = 165)	R group (*n* = 35)	*t*/*χ*^2^	*P*
Age	50.18 ± 3.15	58.39 ± 2.11	14.719	<0.01
Accompanied by family members	128 (77.58)	25 (71.43)	0.606	>0.05
Patient's condition				
I class	78 (47.27)	0	16.663	<0.01
II class	65 (39.40)	5 (14.28)		
III class	12 (7.27)	7 (20.00)		
IV class	10 (6.06)	8 (22.86)		
V class	0	15 (42.86)		
Transfer of escort personnel				
Auxiliary nurse	35 (21.21)	18 (51.34)	16.777	<0.01
Responsible nurse	56 (33.94)	12 (34.29)		
Doctors and responsible nurses	74 (44.85)	5 (14.29)		
Auxiliary ventilation				
Yes	125 (75.76)	10 (28.57)	29.360	<0.01
No	40 (24.24)	25 (71.43)		
Carry medicines and articles				
Yes	153 (92.73)	18 (51.43)	39.724	<0.01
No	12 (7.27)	17 (48.57)		
Carrying line				
Yes	148 (89.70)	18 (51.43)	29.969	<0.01
No	17 (10.30)	17 (48.57)		
Transfer tool				
Flat car	143 (86.67)	8 (22.86)	63.559	<0.01
Wheelchair	22 (13.33)	27 (77.14)		

**Table 3:** Details of each factor assignment.

Factors	Variable name	Variable name
Age	*X*1	≤50 = 0, 51-70 = 1, ≥71 = 2
Patient's condition	*X*2	I class = 0, II class = 1, III class = 2, IV class = 3, V class = 4
Transfer escort personnel	*X*3	Auxiliary nurse = 0, responsible nurse = 1, doctors and responsible nurses = 2
Auxiliary ventilation	*X*4	*Y* = 0, *N* = 1
Transport tool	*X*5	Wheelchair = 0, bicycle = 1
Do not carry drugs and articles	*X*6	*Y* = 0, *N* = 1
Carrying line	*X*7	*Y* = 0, *N* = 1
An accident occurred	*Y*	*Y* = 0, *N* = 1

**Table 4:** Logistic regression analysis of multiple factors affecting in-hospital safe transport in critically ill patients with ICU.

Independent variable name	*β* value	S.E.	Chi-squared value	*P* value	OR value	95% CI
Age	0.813	0.231	12.387	0.001	2.255	1.434-3.546
Patient's condition	0.595	0.134	19.716	0.001	1.813	1.394-2.358
Transfer escort personnel	2.342	1.052	4.956	0.026	10.402	1.323-81.771
Auxiliary ventilation	0.185	0.053	12.184	0.001	1.203	1.085-1.335
Transport tool	2.341	0.942	6.176	0.013	10.392	1.640-65.846
Do not carry drugs and goods	0.923	0.235	15.427	0.001	2.517	1.588-3.989
Carrying line	1.354	0.563	5.784	0.016	3.873	1.285-11.675

## Data Availability

No data were used to support this study.
